The article "Green Finance and Corporate Green Innovation: Based on China's Green Finance Reform and Innovation Pilot Policy" was published in 2022. Journal: J Environ Public Health.

# Green Finance and Corporate Green Innovation: Based on China's Green Finance Reform and Innovation Pilot Policy

**DOI:** 10.1155/2022/1833377

**Published:** 2022-08-03

**Authors:** Shuyu Han, Zuoqian Zhang, Siying Yang

**Affiliations:** ^1^School of Economics, Jilin University, Changchun 130012, China; ^2^Business School, Qingdao University, Qingdao 266071, China; ^3^Centre for China Public Sector Economy Research, Jilin University, Changchun 130012, China

## Abstract

Using data on China's A-share listed enterprises from 2012 to 2019, we investigate the impact of China's green finance reform and innovation pilot (GFRIP) policy on green innovation by the difference-in-difference (DID) method. The results show that the GFRIP policy has a significant role in promoting enterprises' green innovation. Heterogeneity analysis shows that the positive effect of the GFRIP policy on green innovation is only significant for heavily polluting enterprises, large enterprises, state-owned enterprises, and enterprises headquartered in regions with a low level of marketization. Debt financing is an important mechanism for the GFRIP policy to promote corporate green innovation; that is, the GFRIP policy alleviates corporate debt financing constraints and then promotes corporate green innovation. Our study provides theoretical and practical enlightenment for developing countries such as China to deepen reform of the green financial system and promote green innovation.

## 1. Introduction

To catch up economically, China has adopted the development strategy of prioritizing growth and actively promoting industrialization and urbanization to stimulate economic growth, which has caused serious environmental pollution problems. In the context of the global race toward green development and sustainable development, there has been a consensus to establish a green financial system. China has made some progress in developing green finance; however, some financial institutions still have concerns about the risks in the green industry. In 2017, China implemented the green finance reform and innovation pilot (GFRIP) policy in some provinces, which is viewed as a positive step toward developing green finance.

As the mainstay of technological innovation, it is crucial for enterprises to achieve green development in China. To promote enterprises' green innovation, governments generally use environmental regulation tools. However, there is disagreement over the consequences of environmental regulations. On the one hand, well-designed and appropriate environmental regulation policies are considered a contributor to corporate technological innovation [1–4], demonstrating the “Porter hypothesis” [5, 6]. Appropriate environmental regulation can lead to more innovative activities by firms, which increases their productivity and improves firms' profitability in the market. On the other hand, environmental regulations are believed to increase firms' costs and thus inhibit their technological innovation [7, 8]. In addition to environmental regulations, debt financing is essential for green innovation. Enterprises' innovative activities may face financing constraints [9–11]. Environmental regulations may affect the innovation activities of enterprises by easing or decreasing financing constraints.

The article "Green Finance and Corporate Green Innovation: Based on China's Green Finance Reform and Innovation Pilot Policy" was published in 2022. Journal: J Environ Public Health.

The Chinese government attaches great importance to green finance's contribution to the economy. Green finance policies can realize the optimal allocation of financial resources, which is an important exploration for China to promote the development of a green economy by using market instruments such as financial supervision. The GFRIP policy complements traditional environmental regulations. The Chinese government decided to select five provinces (regions) as the first batch of pilots for the GFRIP policy with local characteristics in June 2017, including Zhejiang Province, Jiangxi Province, Guizhou Province, Xinjiang Autonomous Region, and Guangdong Province. Under the guidance of unified macro policies, these regions have actively explored green financial standards, products, and services. Green financial policies with different characteristics have effectively guided the optimal allocation of financial resources; that is, green environmental protection projects have received more fund supplies, while heavily polluting firms (HPFs) are facing increasingly serious financing constraints.

Enterprises need continuous and stable financial support to achieve green innovation. Green finance policies promote the redistribution of financial resources among enterprises by means of strict audit conditions and credit quota management. The Porter hypothesis assumes that HPFs have a stronger incentive than non-heavily polluting firms (non-HPFs) to innovate to increase the “green” content of their products. It is more urgent for HPFs to eliminate the adverse effects of financial regulations on their business. An increasing number of developing countries are promoting green finance and implementing new measures to support green finance with the goal of supporting the sustainable development of enterprises. China has actively issued green bonds and green credit to support the green innovation of enterprises. However, enterprise green innovation and green investment are characterized by longer investment cycles, uncertain income, and imperfect information disclosure. This study reveals the impact of the GFRIP policy on enterprise green innovation. How does the GFRIP policy impact green innovation, and does it have different impacts on different kinds of enterprises? How does the GFRIP policy affect enterprises' green innovation? This study explores, for the first time, the effect of the GFRIP policy and the differences of its impacts and mechanisms among different enterprises using data on China's listed companies. We believe that this study has important theoretical and practical significance for green financial innovation, green financial reform pilot experiments in developing countries, and promoting the green development of enterprises.

The article "Green Finance and Corporate Green Innovation: Based on China's Green Finance Reform and Innovation Pilot Policy" was published in 2022. Journal: J Environ Public Health.

Our research contributes to the current literature on two levels. First, this research complements the existing research into the economic effects of environmental regulations. The existing research on environmental policies focuses mainly on traditional environmental policies, including command and control regulations and market-oriented instruments, such as mandatory emission reduction targets imposed by enterprises and carbon emission trading. The GFRIP policy is a special environmental regulation policy. There is a lack of research on this policy's microeconomic effect and enterprises' innovation behavior. The study analyzes the impact of the GFRIP policy on green innovation and concludes that the policy positively impacts enterprises' green innovation by applying the DID model. Second, this paper provides a new perspective for related research on the GFRIP policy. We analyze the GFRIP policy from the point of view of enterprise innovation and provide more micro evidence for green finance policies. One of the objectives of the GFRIP policy is to promote the green transformation of enterprises and sustainable development. This study confirms the positive effect of the GFRIP policy on enterprises' green development and provides guidance for developing countries that are actively exploring the development of green finance.

## 2. Literature Review

Early research in this area focused on the impact of green financing policies and factors affecting green innovation in enterprises. Green finance includes a range of financial instruments and services, such as green credit, green bonds, green funds, fiscal policy, and green insurance. The Green Credit Guidelines issued in 2012 clearly defined the standards and principles of green credit policies of financial institutions. Liu, Wang, and Kai found that China's Green Credit Guidelines significantly reduced the debt financing of HPFs [12]. Green credit policy truly does have a “reward” effect for non-“two-high and one-high” enterprises and a “penalty” effect for “two-high and one-high” enterprises. According to Hao et al. [13], green credit policy has a favorable impact on heavy polluters in more market-oriented regions, particularly in developing countries. The influence of the green credit policy on HPFs is significantly positive, and this impact occurs mainly through increased credit restrictions [14]. Companies can improve their environmental performance by issuing green bonds, which has a beneficial effect on the company's stock value [15]. However, corporate green bonds do not carry a significant premium and benefit existing shareholders only [16]. Some studies examine the impact of green finance policies from the perspective of the main implementers of the policies. Green credit is effective in improving the credit risk management and core competitiveness of banks [17]. However, it has also been argued that the current low premium for corporate green bonds is not sufficient to convince investors to increase their support for the green bond market [18]. Current studies focus on single financial instruments. Relatively few studies evaluate and examine the comprehensive policy of green finance. Existing studies relating to the comprehensive policy of green finance focus mainly on the relationship between Tobin's q-measured value, the regional innovation level, and corporate social responsibility [19–21]. In conclusion, there is a lack of relevant research into green innovation in enterprises.

The article "Green Finance and Corporate Green Innovation: Based on China's Green Finance Reform and Innovation Pilot Policy" was published in 2022. Journal: J Environ Public Health.

Research on green innovation originated in the 1990s and concerns mostly green technological innovation that reduces environmental pollution and utilizes fewer raw resources and energy. The appellation and definition of green technology often vary depending on the topic of study, for example, environmentally friendly technologies, energy-efficient technologies, renewable energy technologies, and eco-innovations. The World Intellectual Property Organization (WIPO) defines the broadest range of green innovations, including environmentally relevant pollutant disposal and climate change mitigation-related technologies. Hojnik and Ruzzier [22] believed that the main factors influencing firms' green innovation are command-and-control policies, market-oriented policies, and corporate structure. Command-and-control policies include mandatory pollutant monitoring, environmental subsidies, and environmental enforcement [23, 24]; market-oriented policies include environmental rights trading and pollution charges [25, 26]; and the corporate structure involves corporate governance mechanisms and stakeholder pressure [27–30]. Wang and Qi confirmed the role of policy instruments and explored the resulting effects of various policy instruments in different industries and technologies [31]. Enterprises' innovation behavior is also related to their profitability. The profitability of the company can have a positive impact on green product innovation by affecting the legitimacy pressure of the company [32]. There is a positive correlation between environmental innovation and abatement pressures, in which environmental innovation is measured by the number of patents [33]. In addition, enterprise green development and innovation are also related to government decision-making and government behavior [34, 35], for example, the construction of high-tech zones and government-led smart cities in China. Research on the process and the results of enterprise innovation are rich, but research on green finance to promote enterprise green innovation is limited. This study takes the GFRIP policy as a perfect policy test to investigate the effect of green finance on enterprises' green innovation, which enriches relevant research.

The article "Green Finance and Corporate Green Innovation: Based on China's Green Finance Reform and Innovation Pilot Policy" was published in 2022. Journal: J Environ Public Health.

## 3. Theoretical Analysis and Research Hypotheses

Technology innovation is a central component of the new growth theory [36]. Because innovation is long term and uncertain, the financial market allows companies to perform innovative activities. The debt financing of official banks will undoubtedly remain the main source of external financing for companies [37]. Faulkender and Petersen pointed out that capital markets can affect enterprises' capital structure decisions (ability to issue debt) [38]. Nanda and Nicholas revealed that, throughout the Great Recession, the number and quality of corporate patents were hardly influenced by financial difficulty, demonstrating an influential link between credit markets and corporate innovation [39]. Banking competition eases the credit constraints of enterprise innovation [40] and enhances the intensity of enterprise innovation [11]. However, Morck and Nakamura pointed out that the majority of banking-based financial systems hinder the effective flow of external funds into creative industrial technologies [41]. As creditors, banks tend to avoid risks for profitability reasons, and this inherent prejudice in the credit market prevents companies from pursuing innovative activities.

Bank loans are a critical source of capital to invest in company research and development (R&D). According to the social financing scale statistics released by the People's Bank of China, the proportion of bank loans to the total social financing scale was 60.26% at the end of 2020. The traditional financial industry can ignore investment project resources and environmental factors and focus on investment project profitability. Green finance can affect capital flow and promote financial investment from HPFs to high-efficiency industries. If banks and other financial institutions strictly regulate and raise the threshold for obtaining credit support for enterprises, enterprises' financing costs will increase. If the environmental protection information disclosure of enterprises is regarded as a condition for financial institutions to issue loans, the debt financing available to heavily polluting enterprises will be reduced. If financial institutions take the enterprises' environmental performance as a condition for obtaining loans, the debt available to HPFs will be reduced.

The article "Green Finance and Corporate Green Innovation: Based on China's Green Finance Reform and Innovation Pilot Policy" was published in 2022. Journal: J Environ Public Health.

From the perspective of corporate development, corporate innovation has a high rate of failure and requires a large amount of R&D investment. Following the implementation of the GFRIP policy, financial institutions will take environmental performance into account when granting loans. Shareholders will be in turn more willing to encourage managers to strive for corporate green innovation. Limited by the available external R&D investment, enterprises are more willing to drive green development by improving efficiency.

The initial goal of the GFRIP policy is to make the efficient use of financial resources and achieve sustainable economic development. First, financial institutions are encouraged to establish divisions or subbranches to provide diversified financial services. Qualified microfinance and financial leasing companies can participate in green finance. Second, the GFRIP policy encourages the growth of green credit, and the exploration of credit and pledge financing for environmental rights and interests include the following: concession rights, project revenue rights, and sewage rights. The green finance pilot policy provides enterprises within the pilot areas with greater access to multiple sources of financial resources and can alleviate their financing constraints. Third, financial policies support industrial transformation. The GFRIP policy encourages enterprises in pilot areas to obtain financial resources in multiple ways that can alleviate their funding constraints. Hence, the following hypothesis is advanced:

  Hypothesis 1. Companies in the pilot province regions will experience more prominent green innovation performance.

Because of asymmetric information, financial institutions and enterprises face moral hazard and adverse selection problems. Financial resources have been unevenly allocated to different enterprise property rights, scales, and regions for a long time. Enterprises' green development requires financial support. The GFRIP policy will affect enterprises' green development by influencing the redistribution of financial resources. The GFRIP policy is not a specific plan but an overall plan, and pilot regions can develop local specific plans according to regional conditions. This policy will change the flow of financial resources in the region and affect enterprises' green development. The GFRIP policy not only assists firms in achieving energy conservation and emission reduction through provincial technology, but also encourages qualified financial institutions to provide green financial products and services in all aspects to increase the proportion of direct financing for enterprises. Enterprise innovation will take a long time, and green finance policies will provide long-term financial support for enterprise development. Therefore, the GFRIP policy will alleviate corporate debt financing constraints by increasing the scale of debt financing for enterprises, thus facilitating the innovative development of green enterprises. Hence, the following hypothesis is developed:

  Hypothesis 2. The GFRIP policy influences enterprises' green innovation primarily by alleviating debt financing constraints.

The article "Green Finance and Corporate Green Innovation: Based on China's Green Finance Reform and Innovation Pilot Policy" was published in 2022. Journal: J Environ Public Health.

The marginal costs of enterprises with different ownership structures are different, and enterprises will weigh the rising degree of the financing cost. State-owned enterprises (SOEs) often have a good relationship with the local government, so it is easier to obtain implicit government guarantees, and the risk of debt default is relatively low. SOEs have a long life and a stable banking relationship with banks. Therefore, there are great differences between SOEs and non-SOEs in obtaining bank loans. Brandt and Li also argued that non-SOEs are much less likely to obtain loans or that they obtain meager loans and face discriminatory behavior [42]. This difference is observed in companies of different sizes. Technology innovation is usually related to the scale of enterprises. Green innovation requires sufficient R&D, human capital, equipment, technology, and other resources. Large-scale enterprises have obvious advantages in capital, talent, platforms, etc. Small-scale enterprises are unable to maintain high adherence to policies. They make themselves vulnerable if they invest all their resources into one project. The GFRIP policy also has different impacts on enterprises with different pollution levels. Given limited R&D investment, HPFs will improve innovation efficiency to gain debt financing as soon as possible. The regional marketization level also affects the implementation effect of the GFRIP policy. Enterprises in regions with higher marketization levels have multiple financing channels. In addition to bank loans, enterprises' capital sources also include equity financing, green bonds, and other options. Hence, the following hypothesis is developed:

  Hypothesis 3. The GFRIP policy has a more significant impact on green innovation in large-scale enterprises, SOEs, HPFs, and enterprises located in areas with high levels of marketization.

The article "Green Finance and Corporate Green Innovation: Based on China's Green Finance Reform and Innovation Pilot Policy" was published in 2022. Journal: J Environ Public Health.

## 4. Methods

### 4.1. Data Source

The data for this paper have two main sources: (1) data on corporate green innovation. In 2010, the WIPO established an online application to query environmental protection patents, namely, the “International Patent Classification Green List,” which classifies green patents into seven broad categories. Data on corporate innovation in this study were obtained primarily from the Chinese Research Data Services Platform (CNRDS) database, which adheres to the World Intellectual Property Organization's green patent standard and comprehensively sorts and screens patents from the China National Intellectual Property Administration and Google Patents to determine the total number of green patent applications filed, as well as a detailed breakdown of grants granted to Chinese A-share listed companies. (2) Data on company characteristics: the main financial data of listed companies were obtained from the China Stock Market and Accounting Research (CSMAR) database.

This paper's sample is based on Chinese A-share listed companies during the period 2012–2019. A secondary selection is made to guarantee that all publicly available firm data are included by omitting the following: (1) to maintain the comparability of the sample, newly listed companies after 2012 are excluded; (2) due to the significant differences and noncomparability of accounting systems of enterprises of different natures, especially between the financial sector and other industries, the financial indicators of financial enterprises are not comparable to those of other industries, so the sample of listed companies in the financial sector is excluded; (3) companies listed as special treatment (ST and ST^*∗*^) and particular transfer (PT) enterprises firms have been removed due to extraordinary financial performance; and (4) we winsorized continuous variables at the 2% level.

### 4.2. Variables

#### 4.2.1. Explained Variables

Innovation inputs and innovation outputs are widely used in the literature to represent a company's innovation, with innovation inputs indicated mainly by firm R&D and related indicators. As patent data availability increases, and researchers become more devoted to examining patent information, patent data have advantages that make patents important indicators of innovation. Dang and Motohashi pointed out that patents are appropriate indicators of firm innovation [43]. A company's patent data can be divided into patent applications and patent authorizations, which are based on the patent implementation process. It takes a long time from patent application to patent authorization, and the patent may have an impact on the firm's economic performance and technological progress during this period. We use the total number of patent applications for green inventions to quantify the explanatory variable, which is firm's green innovation output (variable *Y*). Specifically, the natural logarithm of the number of indicators above plus 1 is taken to obtain lnPatent.

The article "Green Finance and Corporate Green Innovation: Based on China's Green Finance Reform and Innovation Pilot Policy" was published in 2022. Journal: J Environ Public Health.

#### 4.2.2. Independent Variable

The interaction term between Treat_*i*_ and Policy_*t*_ is the independent variable, where both Treat_*i*_ and Policy_*t*_ are dummy variables. The five provinces (regions) implementing the GFRIP policy were classified as the experimental group, whereas the control group consisted of the remaining provinces (regions). The GFRIP policy is designed as a dummy variable that is allocated a value of 0 before policy implementation, which corresponds to 2017 and earlier; however, the years following policy implementation are assigned a value of 1. We can effectively identify and quantify policy effects by focusing on the coefficient of the interaction term Treat_*i*_ × Policy_*t*_.

#### 4.2.3. Control Variables

We took into account the following variables as control variables on the basis of the literature [14, 35, 44]. The control variables are described as follows: (1) asset: enterprise size is indicated by enterprises' total assets. Firm size is an important factor influencing firm innovation [45]. Larger organizations consistently invest in research and development and have a better success rate with innovation. (2) ROA: ROA is used to estimate the amount of net profit generated per unit of asset [19]. ROA represents the profitability of a company; companies with higher profitability have a greater willingness and ability to invest in innovation activities. (3) Debt: debt is defined as the ratio of a firm's total liabilities to total assets, which reflects the firm's leverage level. Corporate debt reflects the assessment of the company's creditworthiness by the market [46]. A moderately indebted operation may allow a firm to have more funds available for R&D innovation. (4) Tobin's Q: Tobin's Q represents a company's comparative performance. A higher Tobin's Q indicates that the company creates more social wealth and has a higher sense of innovation.

(5) Capital: capital is the ratio of total assets to revenue and represents a firm's reliance on capital investment. Equipment and technology are more important to more capital-intensive firms, which are likely to place greater emphasis on corporate innovation. (6) Largest: companies' organizational structure has a significant impact on operating performance and innovative behavior. Largest is the percentage of largest shareholder shares [47]. (7) Cash: cash demand for corporate R&D will increase over time [48]. This variable represents the ratio of cash and cash equivalents closing balance to current liabilities.

The article "Green Finance and Corporate Green Innovation: Based on China's Green Finance Reform and Innovation Pilot Policy" was published in 2022. Journal: J Environ Public Health.

#### 4.2.4. Mediating Variable

Corporate green innovation often has a long investment cycle, making it more difficult to gain long-term financial support. Whether the GFRIP policy can alleviate the debt financing constraints of enterprises, support their green projects, and influence their green innovation is the key question. The mediating variable is Floan, which is the ratio of the enterprise's long-term borrowing to total assets.

### 4.3. Regression Model

The DID method is commonly utilized to assess the consequences of government policies. The following model was constructed based on the DID method.

Model 1:

(1) $$\begin{array}{c} Y_{it}=\beta_{0}+\beta_{1}\;{\text{Policy}}_{t}+\beta_{2}\;{\text{Treat}}_{i}\times {\text{Policy}}_{t}+\beta_{3}\;{\text{Treat}}_{i}+\gamma \;{\text{Controls}}_{it}+\nu_{t}+\delta_{i}+\varepsilon_{it}. \end{array}$$

*Y*_*it*_ represents a company' green innovation. The GFRIP policy was released in June 2017; considering that there is a certain lag in the implementation of the policy, this paper takes 2017 as the policy time. Policy_*t*_ is a dummy variable for policy implementation, taking a value of 1 for the postimplementation period (after 2017) and 0 for the preimplementation period (2017 and earlier). Taking the GFRIP policy as a quasi-experiment, we assigned the sample companies located in the five provinces (regions) of the experimental area to the experimental group and the others to the control group. *δ*_*i*_ and *ν*_*t*_ denote the industry fixed effect and year fixed effect, respectively. *ε*_*it*_ is the random error term. Our main concern is the interaction term Treat_*i*_ × Policy_*t*_.

## 5. Data Analysis and Results

### 5.1. Descriptive Statistics

Table 1 shows the descriptive statistics for the major variables. The main explanatory variable (lnPatent) has a mean of 0.84, a maximum of 8.285, and a minimum of 0. It is obvious that the number of green invention patents varies widely between companies.

### 5.2. Basic Regression Analysis

As seen in Table 2, there is a strong association between the GFRIP policy and corporate green innovation. In both Columns (1) and (2), the coefficient of Treat_*i*_ × Policy_*t*_ is statistically significantly positive at the 5% level. After controlling for company-level factors such as company size and ROA, the estimated coefficient is 0.084.

The article "Green Finance and Corporate Green Innovation: Based on China's Green Finance Reform and Innovation Pilot Policy" was published in 2022. Journal: J Environ Public Health.

Thus, there is a significant positive correlation between the GFRIP policy and corporate green innovation, which verifies Hypothesis 1. The GFRIP policy is conducive to increasing enterprises' green invention patents in pilot areas. It empowers local governments to adapt their policies to the local context and strengthen green innovations in enterprises through the rational allocation of financial resources. Therefore, the GFRIP policy can play a positive role in supporting enterprises' green transformation.

### 5.3. Reliability Test

#### 5.3.1. Parallel Trend Test

The results of the parallel trend test are meaningful. We conducted the following research to enhance the robustness of our findings. Before the GFRIP policy, green patent applications in different zones should remain largely consistent in terms of time trends. In contrast, after the policy implementation, the parallel trends were broken, and a change in the green innovation trend among enterprises in the pilot provinces (regions) relative to the nonpilot provinces (regions) was observed. The results are shown in Figure 1. The dashed line represents the policy dividing line, and the estimated coefficient of Treat × Policy is apparently not significant to the left of the dashed line, that is, before the policy is implemented, but is strongly positive after implementation. This study passes the parallel trend test.

#### 5.3.2. Placebo Test

A placebo test was conducted to further exclude other unknown factors and ensure that the GFRIP policies led to conclusions. We randomly selected five provinces (regions) from 31 provinces (regions) as the virtual experimental group and assigned the remaining provinces to the virtual control group. The regression was conducted according to the benchmark model, and this randomization process was repeated 500 times. The results are shown in Figure 2, which plots the probability density distribution of the coefficients of the variable Treat_*i*_ × Policy_*t*_ and the corresponding distributions. If the distribution of the estimated coefficients of the variable Treat_*i*_ × Policy_*t*_ is approximately 0, it indicates that no significant factors were omitted from the research design, and the results of the benchmark analysis are more convincing. The coefficient estimates of the virtual regression are all approximately 0, while the benchmark regression's estimates are not included in the virtual regression results. Therefore, the research conclusion is not disturbed by any unobserved missing variables.

The article "Green Finance and Corporate Green Innovation: Based on China's Green Finance Reform and Innovation Pilot Policy" was published in 2022. Journal: J Environ Public Health.

#### 5.3.3. PSM-DID Test

This paper uses propensity score matching with the quantitative difference-in-differences (PSM-DID) method to improve the robustness of the benchmark regression results. We selected Asset, ROA, Debt, Tobin's Q, Capital, Largest, and Cash as covariates and identified variables matching the experimental group in the control group through nearest-neighbor matching within caliper. After matching the covariates, we used the PSM-DID method to test the causal relationship between the GFRIP policy and enterprise green innovation. Column (1) of Table 3 shows the regression results after PSM matching. The coefficient Treat_*i*_ × Policy_*t*_ is positive and significant, so the baseline results according to Model 1 are valid and reliable.

#### 5.3.4. Alternative Measure of Corporate Green Innovation

Next, we sum the number of green invention patent applications and the number of green utility model patent applications and then take the natural logarithm of the above indicator plus 1 to obtain Gpatent2. Then, the explained variables are replaced by the proportion of green patent applications in all patent applications (Gpatent1) and Gpatent2, and the regressions are rerun, as shown in Columns (2) and (3) of Table 3. Even though the explained variables are replaced, the regression results in Table 3 are similar to those of the main regression. The coefficients of Treat_*i*_ × Policy_*t*_ are significantly positive at the levels of 5% and 10%. The above findings justify the selection of lnPatent as the main explained variable and indicate the stability of the findings and the effectiveness of the GFRIP policy to stimulate enterprises' green innovation.

#### 5.3.5. Placebo Test by Replacing Different Policy Times

Considering that the results may be caused by other events prior to the GFRIP policy, this paper uses a placebo test by changing the policy implementation. We assume that policy implementation is moved forward by three years, and we select 2014, 2015, and 2016 as the time of virtual policy implementation. The results are shown in Columns (4)–(6) of Table 3. The coefficient estimates of Treat_*i*_ × Policy_*t*_ are not statistically significant, so the effect of virtual policy impact does not exist. In other words, the effect of the GFRIP policy on corporate green innovation in 2017 is robust, and the estimation results are more reliable.

## 6. Mechanism Analysis

Corporate green innovation activities are often characterized by long payback periods, information asymmetry, and high risk. Under the traditional financial model, it is challenging for enterprises and green projects to obtain long-term financial support, and they face serious problems of maturity mismatch and investment constraints. Green finance is essentially the rationing of financial resources based on environmental constraints. It aims to increase financing capacity and financial support for green projects, reduce financing costs for enterprises, improve the maturity structure of their debt financing, and thus promote their investment and technological innovation in green transformation.

The article "Green Finance and Corporate Green Innovation: Based on China's Green Finance Reform and Innovation Pilot Policy" was published in 2022. Journal: J Environ Public Health.

Next, based on the benchmark analysis, we analyze the mediating effect in greater detail. The mechanism by which green finance policy affects corporate green innovation is examined based on debt financing. This study follows Yang et al. in employing the mediation effect test to construct the following model of the mediation effect [34].

Model 2:

(2) $$\begin{array}{c} M_{it}=\beta_{0}+\alpha \;{\text{Treat}}_{i}\times {\text{Policy}}_{t}+\gamma \;{\text{Controls}}_{it}+\nu_{t}+\delta_{i}+\varepsilon_{it}. \end{array}$$

Model 3:

(3) $$\begin{array}{c} Y_{it}=\beta_{0}+b\;{\text{Treat}}_{i}\times {\text{Policy}}_{t}+cM_{it}+\gamma \;{\text{Controls}}_{it}+\nu_{t}+\delta_{i}+\varepsilon_{it}. \end{array}$$

Variable *M*_*it*_ represents enterprises' debt financing constraints. Regarding the quantification of financing constraints, the KZ index, the WW index, and the SA index are widely used as indicators. Although the KZ index and SA index can also reflect corporate financing constraints, it is more appropriate to use the following indicator. The GFRIP policy has a significant impact on debt financing constraints, and the nonneutrality of long-term debt financing constraints is highlighted in this paper. Following Cao et al., this paper considers that enterprises' green innovation will last for a long time and that firms may be more inclined to use long-term debt obtained from financial institutions for innovation [49]. We use the ratio of long-term debt to total assets to present variable *M*_*it*_, denoted as Floan. The other variables are consistent with the previous section. The mediators of the debt financing constraints of enterprises must be reflected in two aspects. First, Model (2) is introduced to test the relationship between the mediating variables and green finance pilot policy, that is, whether the implementation of the green finance pilot policy affects enterprises' debt financing, which is determined by whether the coefficient of Treat_*i*_ × Policy_*t*_ is significant. Second, the coefficient *b* in Model (3) will be smaller than the coefficient *β*_2_ in Model (1).

Table 4 shows the regression results of debt financing constraints as a mediating variable. The estimated results in Columns (2) and (3) are 0.005 and 0.081, respectively. In Columns (1) and (3), the change in the regression coefficient indicates that the mediating effect exists. Compared with enterprises in nonpilot provinces (regions), enterprises in pilot provinces (regions) can obtain a larger scale of long-term debt financing. The GFRIP policy improves enterprises' green innovation by alleviating debt financing constraints. There is no doubt that the GFRIP policy has created more long-term debt for green projects and technological innovation, and more stable sources of financing and optimized capital structure have improved the willingness to carry out green innovation.

The article "Green Finance and Corporate Green Innovation: Based on China's Green Finance Reform and Innovation Pilot Policy" was published in 2022. Journal: J Environ Public Health.

## 7. Further Discussion: Heterogeneity Analysis

### 7.1. Heterogeneity Analysis Based on Enterprise Ownership

Enterprises with different property rights face different financing constraints, which have different effects on corporate green innovation. SOEs have certain advantages in the allocation of financial resources, especially credit resources, while non-SOEs have long faced credit discrimination. This paper runs a grouped regression by enterprise ownership, distinguishing between a subsample of SOEs and non-SOEs. As indicated in Columns (1) and (2) of Table 5, the estimated result of the SOE subsample is positive at the 1% level, whereas the coefficient of the non-SOE subsample is not significant. The impact of the GFRIP policy is affected by enterprises' property rights, and the GFRIP policy has a greater impact on SOEs. On the one hand, enterprise innovation relies more on external financing, and the advantage of SOEs in obtaining financial resources generally increases the proportion of debt financing. On the other hand, China's green finance system started late and is still in the primary stage of development. The promotion of the GFRIP policy is gradually being explored. Green finance may be more effective in supporting green innovation and the green transformation of SOEs. The information is relatively more comprehensive, and the SOEs in the provinces with green finance pilot policies will benefit more. SOEs have higher policy sensitivity and easier access to comprehensive information. Therefore, in the process of gradually promoting green finance policies, we should pay more attention to non-SOEs to improve the overall effect of green finance in promoting enterprises' green transformation.

### 7.2. Heterogeneity Analysis Based on Pollution Levels

Enterprises' innovative behavior can effectively enhance their own environmental performance and green development capability. The GFRIP policy is an important extension and innovation in relation to traditional environmental regulations. It may have different impacts on enterprises with different pollution levels. In 2008, to further refine the classification of heavily polluting industries for environmental verification, the Ministry of Environmental Protection of the People's Republic of China issued the “Management List of Environmental Verification Industries for Listed Companies,” and combined with the guidelines for industry classification of listed companies, we further divide the enterprises into HPFs and non-HPFs. Columns (3) and (4) of Table 5 show that the coefficient of the HPF subsample is significant at the 5% level. The reasons may be as follows: first, financial institutions regard the green performance of enterprises as an important criterion for granting credit after the implementation of the GFRIP policy. The financing threshold will thus be raised in the short term. With limited debt financing, HPFs are more motivated to enhance their green development by improving innovation efficiency. Second, the GFRIP policy aims to achieve industrial green transformation and the coordinated development of the economy and ecology. This policy is a package that includes many subprojects, and different provinces (regions) can develop differentiated plans according to regional circumstances. For example, Guangdong Province supports the green upgrading of equipment and guides financial institutions to focus on supporting the transformation of highly polluting and energy-consuming enterprises, which provides conditions for green innovation in HPFs.

The article "Green Finance and Corporate Green Innovation: Based on China's Green Finance Reform and Innovation Pilot Policy" was published in 2022. Journal: J Environ Public Health.

### 7.3. Heterogeneity Analysis Based on Corporate Size

Enterprise size reflects the degree of concentration of human capital, production materials, and products within the enterprise. The firm efficiency, financing capacity, and internal control of companies of different sizes differ greatly. We divided enterprises into large-scale enterprises and small-scale enterprises according to the 50th percentile of total assets and investigated whether the promotion effect of the GFRIP policy on enterprise green innovation differed among different enterprise sizes. The regression results for different samples are shown in Columns (1) and (2) of Table 6, which show that the GFRIP policy has different effects on different enterprise sizes. The estimated result is significantly positive at the 5% level for large-scale firms and insignificant for small-scale firms. A possible explanation for this result is that large-scale enterprises have more advantages in gaining financial support, and the current green financial system has a more significant incentive effect on large-scale enterprises. In addition, large-scale enterprises have stronger corporate environmental social responsibility, and credit resources introduced by the GFRIP policy will motivate large-scale enterprises to innovate.

The article "Green Finance and Corporate Green Innovation: Based on China's Green Finance Reform and Innovation Pilot Policy" was published in 2022. Journal: J Environ Public Health.

### 7.4. Heterogeneity Analysis Based on Marketization Level

The degree of marketization of a region can increase or limit the financing channels and options for local firms. On the one hand, regions with higher levels of marketization tend to have more developed financial markets, which can improve the debt financing environment faced by firms and induce them to allocate their limited capital to innovative areas with long-term development value. On the other hand, a higher level of marketization can impact corporate innovation by increasing the anchoring effect of investors and optimizing their structure. In regions with lower levels of marketization, firms face limited financing options and may be more influenced by the policies of green finance demonstration zones. This paper uses the ranking of factor market development in the China Sub-Provincial Marketization Index Report (2021) to measure the degree of regional marketization. Based on the median value of the scores, the sample is divided into firms in regions with high marketization levels and firms in regions with low marketization levels. The results of the grouped regressions are shown in Columns (3) and (4) of Table 6. As seen from the results, the positive effect of implementing the green finance pilot policy on firms' green innovation output in regions with high marketization levels is significant at the 1% level.

## 8. Conclusions and Policy Implications

Green innovation is the essential support and chief motivation for green development and is of great significance in protecting the ecological environment. The GFRIP policy is an excellent quasi-experimental case to explore the association between green finance and enterprise green innovation and provides reliable insight for the development of green finance in developing countries. This paper finds that the GFRIP policy increases the green innovation of companies in pilot provinces (regions) more than that of companies in nonpilot provinces (regions). Furthermore, this study verifies the heterogeneous effects of firm pollution level, firm size, enterprise ownership and regional marketization level. The green innovation promotion effect of the GFRIP policy is more significant for SOEs, HPFs, large-scale enterprises, and firms in regions with high marketization levels. The above results show that the GFRIP policy can significantly promote enterprises' green innovation, but after policy promotion, attention should be given to small-scale enterprises and non-SOEs in the future. Our conclusions provide evidence for the implementation and promotion of green finance policy in developing countries.

The article "Green Finance and Corporate Green Innovation: Based on China's Green Finance Reform and Innovation Pilot Policy" was published in 2022. Journal: J Environ Public Health.

The GFRIP policy seeks to enhance the promotion of green economic development and accelerate green innovation. Our findings provide some policy implications for governments and businesses. First, green finance can reduce environmental risks and promote the sustainable development of enterprises by providing diversified financial products and services to guide capital flows. Developing countries should support the diversification of financial instruments, including green bonds, green insurance, and green funds, and realize the coordinated development of green finance in breadth and depth. We should also consider the interests of nonstate-owned and small-scale enterprises in the distribution of financial resources. Commercial banks should, on the one hand, establish a credit management system that facilitates dynamic adjustments and, on the other hand, innovate green credit processes and services to enhance investment efficiency. Financial institutions should invest financial resources in green industries, pay more attention to enterprises' substantive green behavior in the policy implementation process, improve the rational allocation of green resources, and provide more opportunities and capital for HPFs to promote transformation. The government should support the establishment of a diversified green financial system and promote market-oriented green innovation. Second, enterprises should enhance their social responsibility. Enterprises in developing countries often solve micro-CSR issues, which means that real problems such as environmental protection and green governance are ignored [50]. Enterprises can improve their environmental responsibility by disclosing environmental protection information, improving internal governance, and obtaining more financial support from financial institutions to support their green transformation. Furthermore, stakeholders should increase their enthusiasm for ensuring the supervision of environmental decision-making by enterprises to prevent managers from using environmental costs for personal gain and to reduce resource waste caused by inefficient environmental investment. By reducing principal-agent problems and improving investment efficiency, enterprises in developing countries can improve their green innovation and realize green transformation.

## Figures and Tables

**Figure 1:** Results for common trend test.

**Figure 2:** Results of placebo test.

**Table 1:** Descriptive statistics.

Variable	*N*	Mean	SD	Median	Min	Max
lnPatent	18791	0.84	1.31	0.000	0.000	8.285
Policy	19051	0.25	0.43	0.000	0.000	1.000
Treat	19051	0.28	0.45	0.000	0.000	1.000
Size	18789	22.30	1.36	22.152	14.942	28.636
Capital	18804	2.69	2.14	2.027	0.505	11.117
Big	18805	0.34	0.15	0.311	0.104	0.680
Debt	18805	0.45	0.21	0.439	0.072	0.864
Tobin's Q	18244	2.07	1.34	1.596	0.903	7.233
Cash	18805	0.74	1.09	0.347	0.031	5.763
ROA	18805	0.03	0.06	0.030	−0.184	0.152
Floan	19051	0.04	0.07	0.006	0.000	0.301

The article "Green Finance and Corporate Green Innovation: Based on China's Green Finance Reform and Innovation Pilot Policy" was published in 2022. Journal: J Environ Public Health.

**Table 2:** Results of benchmark regression.

Variable	(1)	(2)
	lnPatent	lnPatent
Treat × Policy	0.092^*∗∗*^	0.084^*∗∗*^
	(0.039)	(0.038)
Policy	0.346^*∗∗∗*^	−0.102^*∗∗∗*^
	(0.030)	(0.035)
Treat	−0.118^*∗∗∗*^	−0.075^*∗∗*^
	(0.043)	(0.037)
Size		0.532^*∗∗∗*^
		(0.024)
Capital		−0.029^*∗∗∗*^
		(0.007)
Big		−0.002^*∗*^
		(0.001)
Debt		−0.173^*∗*^
		(0.103)
Tobin's Q		0.117^*∗∗∗*^
		(0.013)
Cash		0.002
		(0.013)
ROA		−0.073
		(0.235)
Constant	0.295	−11.068^*∗∗∗*^
	(0.184)	(0.544)
Year	Yes	Yes
Industry	Yes	Yes
*N*	18775	18216
*R* ^2^	0.179	0.360

*Note*. ^*∗*^*p* < 0.1;^*∗∗*^*p* < 0.05;^*∗∗∗*^*p* < 0.01.

**Table 3:** Robustness test.

Variable	(1)	(2)	(3)	(4)	(5)	(6)
	PSM-DID	Gpatent1	Gpatent2	*t* = 2014	*t* = 2015	*t* = 2016
				lnPatent	lnPatent	lnPatent
Treat × Policy_*t*_	0.076^*∗∗*^	0.087^*∗∗*^	0.043^*∗*^	0.040	0.024	0.033
	(0.037)	(0.036)	(0.026)	(0.033)	(0.033)	(0.034)
Size	0.535^*∗∗∗*^	0.349^*∗∗∗*^	0.176^*∗∗∗*^	0.311^*∗∗∗*^	0.311^*∗∗∗*^	0.311^*∗∗∗*^
	(0.024)	(0.029)	(0.020)	(0.029)	(0.029)	(0.029)
Capital	−0.029^*∗∗∗*^	−0.011^*∗*^	−0.006	−0.010	−0.010	−0.010
	(0.007)	(0.007)	(0.004)	(0.007)	(0.007)	(0.007)
Big	−0.002	−0.003^*∗*^	−0.001	−0.002	−0.002	−0.002
	(0.001)	(0.002)	(0.001)	(0.002)	(0.002)	(0.002)
Debt	−0.191^*∗*^	−0.060	0.065	−0.123	−0.122	−0.123
	(0.104)	(0.096)	(0.066)	(0.096)	(0.096)	(0.096)
Tobin's Q	0.113^*∗∗∗*^	0.178^*∗∗∗*^	0.113^*∗∗∗*^	0.026^*∗∗∗*^	0.026^*∗∗∗*^	0.026^*∗∗∗*^
	(0.013)	(0.059)	(0.036)	(0.009)	(0.009)	(0.009)
Cash	0.001	−0.005	0.005	0.001	0.001	0.001
	(0.013)	(0.011)	(0.008)	(0.010)	(0.010)	(0.010)
ROA	−0.089	1.756	0.021	−0.166	−0.166	−0.164
	(0.234)	(1.196)	(0.809)	(0.173)	(0.173)	(0.173)
Constant	−11.143^*∗∗∗*^	−6.752^*∗∗∗*^	−3.442^*∗∗∗*^	−6.100^*∗∗∗*^	−6.102^*∗∗∗*^	−6.099^*∗∗∗*^
	(0.549)	(0.640)	(0.435)	(0.646)	(0.647)	(0.647)
Year	Yes	Yes	Yes	Yes	Yes	Yes
Industry	Yes	Yes	Yes	Yes	Yes	Yes
*N*	17797	18287	18287	17889	17889	17889
*R* ^2^	0.361	0.129	0.117	0.105	0.105	0.105

*Note*. ^*∗*^*p* < 0.1;^*∗∗*^*p* < 0.05;^*∗∗∗*^*p* < 0.01.

**Table 4:** Regression results of the mediating effect of debt financing.

Variable	(1)	(2)	(3)
	lnPatent	Floan	lnPatent
Treat × Policy	0.084^*∗∗*^	0.005^*∗∗*^	0.081^*∗∗*^
	(0.038)	(0.002)	(0.036)
Floan			−0.494^*∗∗∗*^
			(0.187)
Constant	−11.068^*∗∗∗*^	0.047^*∗∗∗*^	−7.840^*∗∗∗*^
	(0.544)	(0.000)	(0.555)
Controls	YES	YES	YES
Year	YES	YES	YES
Industry	YES	YES	YES
*N*	18216	18805	18216
*R* ^2^	0.360	0.001	0.086

*Note*. ^*∗*^*p* < 0.1;^*∗∗*^*p* < 0.05;^*∗∗∗*^*p* < 0.01.

The article "Green Finance and Corporate Green Innovation: Based on China's Green Finance Reform and Innovation Pilot Policy" was published in 2022. Journal: J Environ Public Health.

**Table 5:** Heterogeneity analysis results I.

Variable	(1)	(2)	(3)	(4)
	SOEs	Non-SOEs	HPFs	Non-HPFs
	lnPatent	lnPatent	lnPatent	lnPatent
Treat × Policy	0.129^*∗∗∗*^	0.081	0.131^*∗∗*^	0.058
	(0.049)	(0.049)	(0.063)	(0.045)
Size	0.403^*∗∗∗*^	0.458^*∗∗∗*^	0.468^*∗∗∗*^	−0.151^*∗∗∗*^
	(0.031)	(0.033)	(0.036)	(0.046)
Capital	−0.020^*∗*^	−0.012	−0.030^*∗∗*^	−0.096^*∗∗*^
	(0.010)	(0.009)	(0.012)	(0.049)
Big	−0.005^*∗∗∗*^	−0.005^*∗∗∗*^	−0.001	−0.002
	(0.002)	(0.002)	(0.002)	(0.001)
Debt	−0.161	−0.043	−0.254	−0.158
	(0.130)	(0.123)	(0.161)	(0.134)
Tobin's Q	0.026^*∗*^	0.090^*∗∗∗*^	0.090^*∗∗∗*^	0.129^*∗∗∗*^
	(0.016)	(0.016)	(0.020)	(0.018)
Cash	−0.038^*∗*^	0.002	0.000	0.000
	(0.021)	(0.014)	(0.018)	(0.017)
ROA	−0.324	0.199	−0.201	0.002
	(0.278)	(0.270)	(0.345)	(0.305)
Constant	−8.044^*∗∗∗*^	−8.783^*∗∗∗*^	−10.139^*∗∗∗*^	−11.878^*∗∗∗*^
	(0.695)	(0.764)	(0.776)	(0.687)
Year	Yes	Yes	Yes	Yes
Industry	Yes	Yes	Yes	Yes
*N*	7225	9322	6286	11518
*R* ^2^	0.123	0.284	0.265	0.392

*Note.* ^*∗*^ *p* < 0.1;^*∗∗*^*p* < 0.05;^*∗∗∗*^*p* < 0.01.

**Table 6:** Heterogeneity analysis results II.

Variable	(1)	(2)	(3)	(4)
	Small-scale firms	Large-scale firms	Market < *p*50	Market > *p*50
	lnPatent	lnPatent	lnPatent	lnPatent
Treat × Policy	0.057	0.101^*∗∗*^	0.107	0.140^*∗∗∗*^
	(0.056)	(0.046)	(0.095)	(0.033)
Size	0.418^*∗∗∗*^	0.381^*∗∗∗*^	0.472^*∗∗∗*^	0.413^*∗∗∗*^
	(0.034)	(0.036)	(0.053)	(0.026)
Capital	−0.002	−0.011	−0.016	−0.007
	(0.012)	(0.008)	(0.014)	(0.008)
Big	−0.008^*∗∗∗*^	−0.001	−0.006^*∗*^	−0.005^*∗∗∗*^
	(0.002)	(0.002)	(0.003)	(0.002)
Debt	−0.268	−0.255^*∗∗*^	−0.394^*∗∗*^	−0.266^*∗∗*^
	(0.176)	(0.113)	(0.190)	(0.112)
Tobin's Q	0.053^*∗∗∗*^	0.014^*∗*^	0.015	0.026^*∗∗∗*^
	(0.020)	(0.008)	(0.016)	(0.008)
Cash	−0.002	−0.024^*∗∗*^	−0.053^*∗∗*^	−0.009
	(0.024)	(0.011)	(0.022)	(0.011)
ROA	0.048	−0.595^*∗∗∗*^	−0.610^*∗*^	−0.308
	(0.338)	(0.196)	(0.356)	(0.194)
Constant	−8.204^*∗∗∗*^	−7.205^*∗∗∗*^	−9.362^*∗∗∗*^	−8.088^*∗∗∗*^
	(0.801)	(0.765)	(1.202)	(0.604)
Year	Yes	Yes	Yes	Yes
Industry	Yes	Yes	Yes	Yes
*N*	8768	8632	4041	13763
*R* ^2^	0.107	0.065	0.090	0.085

*Note*. ^*∗*^*p* < 0.1;^*∗∗*^*p* < 0.05;^*∗∗∗*^*p* < 0.01.

## Data Availability

Data supporting the findings of this study are available from the corresponding author upon reasonable request.
